The article "Electron Microscope Observation of Acupuncture and Nerve Repair in the Treatment of Peripheral Facial Paralysis" was retracted in 2023. Reasons: signs of a paper mill; suspected computer-generated content; unreliable results or conclusions; lack of ethics approval or compliance.

# Electron Microscope Observation of Acupuncture and Nerve Repair in the Treatment of Peripheral Facial Paralysis

**DOI:** 10.1155/2022/5432223

**Published:** 2022-07-13

**Authors:** Zhenggen Shan

**Affiliations:** Sichuan Vocational College of Health and Rehabilitation, Zigong, Sichuan, China

## Abstract

The repair of peripheral facial paralysis is a long-term problem in neurosurgery, and nerve repair is often needed. Due to the high differentiation of nerve tissue and the slow regeneration of peripheral nerve fibers, the repair effect after peripheral nerve injury is not ideal. In recent years, studies have found that the inflammatory response after peripheral nerve injury also has an important impact on the repair of peripheral nerve defects. This study depends on the utilization of traditional needle therapy in the treatment of fringe facial loss of motion, and the clinical adequacy of needle therapy in addition to nerve fix in the intense period of fringe facial loss of motion was seen with an electron magnifying lens. Endeavor to give significant exploration results to the clinical treatment of fringe facial loss of motion gives a straightforward, simple, protected, and successful new treatment innovation for the clinical treatment of the infection and enriches the treatment plan for peripheral facial paralysis. Transmission electron microscopy observations showed that 21 days after the artificial nerve was repaired, the nerve injury showed different degrees of recovery, and the myelin sheath was forming and gradually wrapping the new axons, which was similar to the catheter group (NC) and hydrogel group (HC). In contrast, the myelin layer of the fibroblast group (FHC) is more obvious, and the repair effect is better. In the maintenance of fringe nerve surrenders, irritation is an unavoidable interaction, and moderate needle therapy is useful to advance the maintenance of fringe nerve abandons. Talking about the law of nerve fix reaction in fringe nerve imperfection fix is helpful to the examination of fringe nerve deformity fix. Tests have shown that utilizing needle therapy and moxibustion joined with nerve fixes has accomplished great outcomes in the treatment of fringe facial loss of motion, and the patient's recuperation rate has expanded by over 30%.

## 1. Introduction

Fringe facial nerve paralysis (PFP) is additionally called Bell's paralysis, idiopathic facial nerve paralysis, and facial neuritis. It is the reason for fringe facial nerve paralysis, its goal is not clear, and there could be no different side effects and qualities. Modern medicine speculates that the disease may be caused by perifacial paralysis caused by nonspecific inflammation of the facial nerve in the trunk organ. It was first described by Charles Bell in 1821. To commemorate Bell, the descendant doctor William The Gowers was named after Bell. Peripheral facial nerve palsy usually comes on suddenly. Before it starts, the patient may have wind, cold, or fatigue, and there may be pain or fever from the back of the ear to the skin behind the ear bones and cheeks. The affected side may be paralyzed, the nasolabial fold may flatten, and the corners of the mouth may tilt. It is completely different from the healthy side. The wrinkles on the forehead disappear, the eyes are swollen, and the face is dull and numb. Peripheral facial paralysis is called facial neuritis, which is caused by the acute inflammation and edema of the stylomastoid foramen of unknown origin, but 10% to 25% of the patients cannot fully recover due to mistreatment or serious illness and even suffer from severe disease—leaving serious sequelae, causing great harm to the patient's body and mind. Therefore, how to cure facial paralysis at the best time is imminent.

In modern medicine, the cause of peripheral facial nerve palsy is not yet fully understood. Hormone therapy is the main treatment method, but the effect is not very satisfactory. Sun summarized the academic thoughts and clinical experience of Professor Sun Shentian's acupuncture treatment of peripheral facial nerve palsy. According to the different stages of facial paralysis, Professor Sun's treatment plan has its own focus. In the acute phase, Professor Sun emphasized the importance of standardized western medicine treatment and made recommendations for early acupuncture treatment. Treatment is mainly focused on dispelling wind and cold, promoting blood circulation, and dredging collaterals. In the rehabilitation phase, Professor Sun emphasized the “needle removal method” and repeated transcranial acupuncture according to the functional direction of the cerebral cortex. In the sequelae stage, Professor Sun emphasized the value of regulating thoughts. During the treatment, Professor Sun paid great attention to flexible acupuncture point selection, repeated transcranial acupuncture, “needle removal” method, acupoint pressing, and giant needle method, as well as the combined use of electric acupuncture and directional injection. However, the treatment method is too slow to suppress the condition in time [1]. Lv et al. investigated the impact of back rub on quality articulation in rodents with sciatic nerve injury (SNI). They explained the maintenance component of back rub to advance the recuperation of fringe nerve injury. In the joke activity bunch, the right sciatic nerve was uncovered without a brace. The SNI model was laid out on the right leg with sciatic forceps and afterward arbitrarily isolated into SNI gathering and back rub bunch. Seven days in the wake of demonstrating, the back rub group utilized the “Back rub Massage Manipulation Simulator” for treatment consistently. The simulator was used to stimulate the silver gate (BL37) every day. The stimulation force was 4N and the stimulation frequency was every minute. Use each method and each acupuncture point for 1 minute, for a total of 9 minutes. However, this method has sequelae to the patient and needs to be treated according to the situation [2]. Lovaglio AC accepts that fringe nerve and brachial plexus injury typically prompts extreme harm to the impacted appendage. The rate of neuropathic torment is exceptionally high, particularly on account of cervical root separation, as high as 95% of cases. Neuropathic torment is brought about by harm to the somatosensory framework, and its ongoing advancement process relies upon the harm that influences the encompassing and focal sensory system. The treatment of these agonies is extremely convoluted and should be finished by a multidisciplinary group. From the first-line pharmacological treatment (Such as tricyclic antidepressants and calcium channel ligands) start with physical and word-related treatment, transcutaneous electrical feeling, and mental help. For patients who experience issues getting introductory treatment, a few neurosurgery choices are accessible, including nerve decompression or reproduction and removal/molding systems. Yet, this will defer the ideal time of patient treatment, and the condition might change [3].

This article depends on the utilization of needle therapy and treatment of fringe facial loss of motion and the utilization of an electron magnifying instrument to screen the clinical impacts of needle therapy and nerve fix in the intense period of fringe facial loss of motion [4]. Aiming at the research on limbic facial nerve palsy, and comparing many treatment methods, find out the advantages and disadvantages of different treatment methods, accumulate experience, and make more contributions to traditional Chinese medicine. It gives significant exploration results to the treatment of intense fringe facial loss of motion and gives a solid premise to bed rest. After the beginning of fringe facial nerve paralysis, the facial nerve is compacted in the intense stage, and the facial nerve tube is ischemia and hypoxia, bringing about degeneration, edema, and even demyelination. The more pressure on the facial nerve, the more degeneration, and it is difficult to recover. The degree of facial nerve injury determines the severity and prognosis of facial paralysis [5, 6]. Early consultation and timely intervention are protective factors in restoring facial nerve palsy. Therefore, treatment in the acute phase is very important. The research on the repair of peripheral facial paralysis is a convenient reference for future medical development.

## 2. Treatment of Peripheral Facial Paralysis

Modern medicine believes that the treatment of peripheral facial paralysis through the functional recovery of the facial nerve is the most scientific and simple method; since ancient research, TCM has formed a sound TCM theoretical system in the treatment of “slanting eyes and mouth.” The etiology and pathogenesis of this disease have been perfected under the continuous research and exploration of senior Chinese medicine practitioners.

### 2.1. Diagnostic Criteria of Chinese Medicine

Allude to the New Century (Second Edition) course book “Needle therapy and Moxibustion Therapy” (altered by Wang Qicai, China Press of Traditional Chinese Medicine, 2007) [7, 8]:

1. The onset is sudden, usually in winter and summer, and often has a history of cold and cold or pain in the bone behind the ear when some patients first onset;
2. Muscles on the side of the disease are numb and stiff, forehead lines become shallow or disappear, eye fissures become wider, eyes open and tear, nasolabial fold becomes shallow, mouth corners droop and crook to the healthy side;
3. The sick side cannot do actions such as frowning, closing eyes, bulging cheeks, and showing teeth [9, 10].

Inadequate qi and blood classification: more normal in patients with recuperation period or a long course of sickness, appendages languor and shortcoming, pale composition, wooziness, short breath, lethargic discourse, palpitations, perspiring, pale tongue, dainty white fur, slim and frail heartbeat [11, 12].

### 2.2. Western Medicine Diagnostic Criteria

In line with the “Neurology” of Western medicine, the diagnostic criteria for idiopathic facial nerve palsy and facial neuritis:

1. The onset is rapid, and the symptoms of facial nerve palsy often rise to the peak in a short period of time; it is more common on one side;
2. The facial expression muscles of the disease are paralyzed, the forehead lines disappear, the forehead frowning cannot be performed, and the eye fissures become enlarged;
3. When the eyes are closed, the white sclera of the diseased eye is exposed;
4. The nasolabial folds become shallow, the mouth corners droop during static observation, and the mouth corners are skewed toward the healthy side when performing tooth-exposing movements;
5. The sick side often leaks air when doing puffing movements, and food residues are easy to keep on the sick side's gums;
6. In some cases, abnormal taste in the front 2/3 of the tongue, or hyperacusis can be seen;
7. The electromyography is abnormal [13, 14].

### 2.3. Adverse Events and Treatment Methods

1. Needle dizziness: the patient has symptoms such as nausea and vomiting, pale complexion, cold limbs, dizziness, and palpitation, etc., and the needle should be taken immediately, and the patient should be assisted to lie supine with the head low and the feet high, and keep warm [15, 16]. Give patients appropriate warm water orally. Generally recoverable, if the situation is serious, emergency treatment should be taken immediately.
2. Hematoma: local small bruises after needle removal are mostly caused by a small amount of subcutaneous hemorrhage, which usually resolves spontaneously and does not require special treatment. If the bruising area is large and accompanied by local pain and swelling, apply cold compresses to stop the bleeding first, and then slowly rub or apply heat to the local area to dissipate and absorb blood stasis.
3. Scald: the flash tank operation causes small blisters to appear locally. As long as they are not rubbed, they can not be treated, and they can be absorbed naturally. If the blisters are large, the local skin should be strictly disinfected first, and then the blisters should be pierced with a thick needle to release the liquid, and the blisters should be disinfected again and then wrapped with gauze.

### 2.4. Principles of Peripheral Nerve Injury Repair

The main function of nerve fibers is to conduct nerve impulses. The conduction speed of various nerve fibers is different, roughly between 3 and 120 meters per second. Those that transmit nerve impulses from receptors to the central nervous system are called afferent fibers; those that transmit impulses from the central nervous system to effector organs are called efferent fibers. Nerve fibers are the protrusions of neurons, and the neuron cell body is the nutrient center of neurons [17, 18]. Due to injury or other reasons, nerve fibers may be cut out of the cell body, which may cause damage and death. This process is called nerve fiber ulcer. At this point, the peripheral shaft and myelin sheath and some proximal shafts first expand, then collapse, and collapse into fragments and droplets called plaques. Protective inflammation is an important part of innate immunity after peripheral nerve injury, and it is a necessary step to promote wound healing and functional reconstruction. After 3 days of nerve injury, fibroblasts migrate from a calm state to a migrating state and gradually migrate to the center of the wound. At the same time, they multiply rapidly and synthesize a large amount of collagen and fibronectin. On the 14th day after the injury, fibroblasts transform into a contractile phenotype to induce various cytokines, namely myofibroblasts, and the extracellular matrix is regulated by integrins on the surface of fibroblasts, leading to wound contraction [19, 20]. After wound healing, the number of myofibroblasts decreases due to programmed death. On the one hand, fibroblasts multiply, synthesize, and secrete a large amount of extracellular matrix to fill tissue defects. On the other hand, the extracellular matrix acts as a framework and binding role. It regulates the migration, differentiation, and proliferation of fibroblasts and also acts as a “reservoir” for regulating fibroblasts through local accumulation and release of growth factors. During the regeneration of peripheral nerves, fibroblasts multiply and migrate to fill the defect. Then, they migrate Schwann cells from the proximal end to the distal end through signal transduction pathways and finally make the axons lower than the Schwann cells. The guide extended to the end [21].

As shown in Figure 1, regeneration of nerve fibers usually occurs 2–3 weeks after injury. The Nissl body corresponding to the damaged nerve fiber gradually returned to its normal shape, the nucleus returned to the center, the proximal end of the damaged nerve axis was connected and oriented to the cell body, and many steps grew on the edge. Some of these young shoots passed through the tissue gap in the injury, grew long distances along with Schwann cells, and finally reached the original tissues and organs [22, 23]. Some young shoots penetrate the connective tissue of the nerve and form neuroma, while the rest of the young shoots degenerate or disappear. The axial shoots growing along Schwann cells continue to thicken, myelin sheath gradually forms, and the function of nerve fibers gradually recovers. At that time, the regeneration process of nerve fibers is also completed in advance.

## 3. Peripheral Nerve Injury Repair Correlation Experiment

### 3.1. Determination of Pla/Go Conductivity

The electrical conductivity was analyzed by measuring the volume resistivity of the fiber membrane, and the volume resistivity of the PLA/GO electrospun fiber membrane was tested with a four-point probe measuring instrument. At room temperature, test each group of samples five times and calculate the average value. The calculation formula (1) of the volume resistivity (*R*) of PLA/GO is as follows:

(1) $$\begin{array}{c} R=0.628\times \frac{V}{I}\times \text{Thick.Correct}\times \text{Temp.Correct}\times \text{Edge.Correct}. \end{array}$$

In the formula, V/I is the surface resistance of the PLA/GO electrospun fiber membrane, Thick.Correct is the thickness correction coefficient, Temp.Correct is the temperature correction coefficient, and Edge.Correct is the side length correction coefficient.

Take out the fiber membrane soaked in ethanol, weigh the mass of the remaining pycnometer and ethanol as M3, measure each sample 5 times in parallel, and take the average value. The porosity is shown in the following formula (2):

(2) $$\begin{array}{c} \text{porosity}\left(\text{\%}\right)=\frac{M_{2}-M_{3}-M_{0}}{M_{1}-M_{3}\times 100\%}. \end{array}$$

According to the experimental load and the size of the fiber membrane, the corresponding stress value is calculated, and the stress-strain curve can be obtained from the load-deformation curve. Each valid sample was tested in parallel 5 times, and the average value was taken [24, 25]. The tensile strength (MPa) is calculated according to formula (2):

(3) $$\begin{array}{c} \delta =\frac{F}{b\times d}. \end{array}$$

The elongation at break (%) is calculated as shown in formula (3):

(4) $$\begin{array}{c} \varepsilon =\frac{L-L_{0}}{L_{0}}. \end{array}$$

Because the pH environment exceeds a certain range of pH, the degradation of the fiber membrane in the solution is affected. In order to ensure that the pH value of the solution environment is around 7.4, new PBS solution needs to be added regularly, twice a week. Calculate as follows to obtain the weight loss rate of the fiber membrane:

(5) $$\begin{array}{c} W\left(\%\right)=\frac{\left(W_{0}-W_{1}\right)}{W_{0}}\times 100\%, \end{array}$$

where *W* is the weight loss rate; the initial mass of W_0_ fiber membrane [26]; the mass of W_1_ after different degradation times. According to formula (4), calculate the cumulative release percentage of NGF and draw the release curve.

(6) $$\begin{array}{c} Q\left(\%\right)=\frac{V_{0}\times C_{t}+V\times \sum_{n-1}^{t-1}C}{M}. \end{array}$$

### 3.2. Electron Microscope Observation Method

Electron microscopy is an instrument that replaces light beams and optical lenses with electron beams and electron lenses based on the principles of electron optics to image the fine structures of matter under very high magnification. In recent years, the research and manufacture of electron microscopes have made great progress: on the one hand, the resolution of electron microscopes has been continuously improved, the point resolution of transmission electron microscopes has reached 0.2–0.3 nm, and the lattice resolution has reached about 0.1 nm, people have been able to directly observe atomic images; on the other hand, in addition to transmission electron microscopes, a variety of electron microscopes have been developed, such as scanning electron microscopes, analytical electron microscopes, etc. Silicon is anisotropic during wet etching. As shown in Figure 2, the schematic diagrams of the etching of silicon with (100) crystal orientation and (110) crystal orientation in KOH solution are shown, respectively.

When the size of (100) crystal phase silicon is small, it will automatically stop on the (111) crystal plane after KOH etching, forming a pyramid shape. The relationship between the etching depth and the shorter side length of the uncovered silicon is shown in the formula [27]:

(7) $$\begin{array}{c} h=\frac{L}{2}*TG\left(63.2{}^{\circ}\right), \end{array}$$

where *h* is the depth of etching and *L* is the shorter side length of the exposed surface. When the silicon is etched through, the relationship between the etched size formed on the other side of the silicon and the size not covered by silicon nitride is as shown in the formula:

(8) $$\begin{array}{c} w=W-2H*ctg\left(63.7{}^{\circ}\right). \end{array}$$

The observation of the Coulomb blockade effect generally needs to meet two conditions.

(9) $$\begin{array}{c} R_{T}>R_{K}-c, \end{array}$$

(10) $$\begin{array}{c} \frac{e^{2}}{C\gg kT}. \end{array}$$

Here, C is the tunneling junction capacitance and T is the measured temperature. The smaller the junction capacitance C, the higher the measurement temperature T, k is Boltzmann's constant, and T is the temperature of the nanometer point [28, 29]. When the size of nanomaterials decreases, the self-capacitance of nanomaterials also decreases, which means that it is easier to observe the Coulomb blockade.

(11) $$\begin{array}{c} \frac{77k\ll e^{2}}{C\ll 300k}. \end{array}$$

For the spherical nanodots of InAs, the capacitance of the nanodots is as follows:

(12) $$\begin{array}{c} C=\pi \varepsilon_{r}\varepsilon_{0}r-200k+\frac{cd}{\sum_{R}t-3}. \end{array}$$

The calculation shows that when the 10 nm nanodots of InAs nanodots exhibit Coulomb blockage at liquid nitrogen temperature, the Coulomb blockage phenomenon will disappear at room temperature.

## 4. Effect of Acupuncture on Peripheral Facial Paralysis

### 4.1. H-B Facial Nerve Classification before and after Treatment

Before treatment, the two groups were analyzed by Ridit, *t* = 0.587, *P*=0.560 > 0.05, indicating that the difference between the two groups before treatment was not significant; after treatment, the two groups were analyzed by Ridit, *t* = −0.583, *P*=0.012 < 0.05, indicating that after treatment, there is a statistical difference between the two groups; in the comparison of the treatment group before and after treatment, through Ridit analysis, it can be obtained: *t* = 2.122, *P*=0.044 < 0.05, indicating that the effect of the treatment group before and after treatment is obvious, and the difference can be considered as statistical significance. In the comparison between before and after treatment in the control group, Ridit analysis showed: *t* = 2.618, *P*=0.019 < 0.05, indicating that the HB facial nerve grading of the treatment group was significantly different before and after treatment. It can be seen from the results of statistical data analysis that during the course of treatment, the HB classification changes of the treatment group and the control group before and after treatment were more obvious, and the treatment effect of the treatment group (acupuncture + acupuncture) was obvious, as shown in Table 1.

After all the treatment courses are completed, through the comparison of various evaluation indicators and after statistical technical analysis, it is determined that the evaluation indicators are statistically significant, and it is concluded that the scoring results after treatment have significant changes compared with those before treatment, as shown in Figure 3.

After the completion of all treatment courses, through the comparison of various evaluation indexes and the statistical technical analysis, it is determined that the evaluation indexes are statistically significant. Furthermore, it is reasoned that the scoring results after treatment have massive changes contrasted and those before treatment. To be specific (*P* < 0.05), looking at the treatment bunch (needle therapy + needle therapy) and the benchmark group (needle therapy), the treatment gathering's recuperation rate is more huge than the benchmark group; the treatment bunch (needle therapy + needle therapy) and the benchmark group (needle therapy) all out compared with the powerful rate, the successful pace of the treatment bunch is more critical than that of the benchmark group. Through the examination of trial information, it tends to be seen that needle therapy joined with needle therapy treatment is more successful in the treatment of patients with “fringe facial loss of motion” in the recuperation time frame, as shown in Figure 4.

The fix rate and successful pace of the treatment bunch were 60.00% and 83.33% separately; the fix rate and compelling pace of the benchmark group were 46.67% and 73.33%, individually; the fix rate and powerful pace of the treatment bunch were more huge than those of the benchmark group. The position total test information examination shows that 2w = 19.733, *P* = 0.006 < 0.01; there is a tremendous distinction; this indicates that this experiment has research significance.

As shown in Table 2, the treatment process of the two groups of cases progressed smoothly. Another 5 people had a certain psychological rejection of acupuncture during the treatment process, which had a certain impact on the treatment effect, but did not have much impact on the overall treatment effect, including 3 cases in the treatment group and 2 cases in the control group.

The comparison of the curative effects of the three groups is shown in Figure 5. Through moxibustion on acupoints and local points, the vascular permeability of the local skin is increased and the pores are expanded, thereby promoting the absorption of drugs and giving full play to the curative effect of drugs. Combining the functions of acupoints, it can harmonize internal and external effects, improve the body's immune function, promote the elimination of local inflammatory factors, accelerate the absorption of inflammatory exudate, and promote swelling, pain elimination, and skin lesion recovery. This also reflects the role of traditional Chinese medicine in “strengthening the body and eliminating evils,” which can relieve pain, promote qi and blood circulation, clear heat, relieve fire, expel wind, relieve itching, and reduce swelling. The medicinal thread moxibustion therapy is simple in operation, rigorous in theoretical content, and effective. In a sense, it has the function of auxiliary treatment.

### 4.2. Microscopic Observation of Nerve Recovery Analysis

It is understandable that fibroblasts and Schwann cells are contained in the fibroblast group, but they are also contained in the catheter group and hydrogel group, indicating that the regeneration activity of peripheral nerve injury has been carried out at 14 days. Other cells that do not develop color correspond to the figure. It is guessed that they are red blood cells or inflammatory cells, indicating that the inflammatory response is still going on at this time. There are more fibroblasts and Schwann cells in the fibroblast group than in the catheter group and the hydrogel group, indicating that the fibroblast group has more active cell repair after peripheral nerve injury, and the repair may be faster, as shown in Figure 6.

The normal nerve longitudinal section was used for immunofluorescence staining of the fibroblast marker Fibronectin (green fluorescence) and nuclear DAPI (blue fluorescence). The picture shows that after a normal nerve longitudinal section, clear-textured nerve fibers can be seen. These nerve fibers are composed of neuron axons and outer glial cells (Schwann cells), so only weak fluorescence can be seen. Green fluorescence (Fibronectin, a marker for fibroblasts) can also see obvious nuclei in nerve fibers [30, 31]. Compared with the fluorescence intensity of normal nerve longitudinal section Schwann cells, the fluorescence intensity of Schwann cells in the hydrogel group is weaker, and the fluorescence intensity of normal nerve Schwann cells is stronger. This shows that the Schwann cells in the hydrogel group are less than those in the normal nerves, and the proximal and tube wall fibroblasts in the hydrogel group are slightly more than those in the normal nerves. There was little difference in the number of fibroblasts in the distal and normal nerves in the group.

The nervous system is the most important tissue system in the human body. It regulates the sensation and movement of various parts of the body. Therefore, once the nerves are damaged, the normal functions of various organs will also be affected. As shown in Figure 7, with the help of light microscopy or electron microscopy technology, we can visually observe from the morphology that Schwann cells guide axon regeneration from dedifferentiation, proliferation, migration, and then differentiation and sparing axons after nerve injury. Hence, behind these interesting biological phenomena, which molecules are involved? In order to understand this complex gene network in depth, we still use the above three different types of rat sciatic nerve defect/repair models, namely the Sca group, the TENG group, and the Auto group. At the same time, a sham operation (Sham) group is set up to eliminate surgical factors. Interference, at different time points after surgery (1 d, 4 d, 1 w, 2 w, 3 w, 4 w, 8 w, 12 w), the bridging segment tissues of each group of animals were obtained. In the Sham group, the sciatic nerve at the same position was taken, and the tissue RNA was extracted to perform gene Chip detection. Search for myelin-related genes (including related genes involved in Schwann cell dedifferentiation, proliferation, migration, differentiation, myelination, myelin thickness, etc.) through the IPA (Ingenuity Pathway Analysis) database, and then extract these genes with the chip data Intersection, a total of 383 myelin-related genes were obtained (it may increase after the IPA database is updated); Hierarchical cluster analysis (Hierarchical clustering analysis) was performed on the myelin-related genes at all time points in the Sca, TENG, and Auto groups using bioinformatics analysis tools. Clustering, HCL, or Principal Component Analysis (PCA) analyzes the clustering situation of each group of samples at each time point or the positional relationship in three-dimensional space and conducts gene network analysis on the biological process of remyelination through the IPA database, through the Venn diagram to show the similarities and differences of the molecules involved in each biological process of the Sca, TENG, and Auto groups, and perform immunohistochemistry and PCR verification.

As shown in Table 3, observe the tissue sections of the four groups of regenerated nerves at various time points through a microscope, compare and analyze the regeneration of each group of nerves and the differences between groups, and observe the formation of regenerated nerves and the growth of myelinated nerve fibers. Nikon picture analyzer: each cut arbitrarily chooses 5 fields of view, counts the number of myelinated nerve strands per unit region, and measures the thickness of the myelin sheath of the myelinated nerve. The recuperation of facial nerve work was decided by the inertness of the activity capability of the orbicularis oris muscle, the conduction speed of the recovering nerve, and the sufficiency of the compound neuromuscular activity potential in trial creatures. Use SPSS22.0 statistical analysis software to analyze neuromuscular action potential latency, amplitude, regenerative nerve conduction velocity, number of myelinated nerve fibers, and myelin thickness, etc., use one-way analysis of variance, and then use LSD-*t* test for pairwise analysis. For comparison, the measurement data is expressed as (± *s*), and the test level is *α* = 0.05, *P* < 0.05, the difference is considered to be statistically significant.

As shown in Table 4, the examination between the two gatherings before treatment was not measurably huge (*P* > 0.05), and the correlation between the treatment bunch when treatment *Z* = −5.092, *P* = 0.000 < 0.01; there was a massive distinction. When treatment in the benchmark group, *Z* = −5.090, *P* = 0.000 < 0.01, there is a tremendous contrast. The examination between the two gatherings after treatment was measurably huge (*P* < 0.05). Note: the two gatherings are practically identical after treatment. After treatment, the fringe facial nerve paralysis scale scores of the treatment bunch and the benchmark group are worked on contrasted with before treatment, and there is a distinction in the scores of the fringe facial nerve paralysis scale between the two gatherings.

The neural network abstracts the human brain neuron network from the perspective of information processing, establishes a certain simple model, and forms different networks according to different connection methods. As shown in Figure 8, on the 3rd, 7th, and 14th days of nerve repair, white blood cells, red blood cells, and cells of nonblood cell lines can be observed in each group. These cells have different morphologies. It may be fibroblasts or Schwann cells. For the group of fibroblasts, since fibroblasts are added to artificial nerves, it is expected that cells of nonblood cell lines can be observed. In the nerve conduit group and the hydrogel group, since no cells were added, cells of nonblood cell lines were observed. Theoretically, these cells may be derived from the distal or proximal end of the recipient sciatic nerve or may be caused by the differentiation of hematopoietic stem cells, which seems to mean that on the third day of artificial nerve repair, nerve defect repair activities have started. At the same time, the appearance of white blood cells indicates that the inflammatory response has started on the third day of artificial nerve repair. The distribution of capillaries in the sciatic nerve is underdeveloped, and material exchange mainly depends on tissue fluid [32]. The appearance of red blood cells indicates that blood is directly involved in the repair of peripheral nerve defects. From the 14th day to the 21st day of artificial nerve repair, the proportion of nonblood-line cells gradually increased, indicating that the repair process of peripheral nerve defects is proceeding more quickly, and a large number of nonblood-line cells are secreted to promote the regeneration of peripheral nerves. The gradual decrease of white blood cells indicates that the intensity of the inflammatory response is gradually weakening. There are fewer white blood cells in the fibroblast group, indicating that the inflammatory response is weaker. From the 21st to the 30th day of nerve repair, nonblood cells increased in the three groups, indicating that nerve regeneration was more vigorous. There was a limited quantity of white platelets in the fibroblast bunch, the nerve channel bunch, and the hydrogel bunch, demonstrating that the provocative response in the fibroblast bunch, the nerve conduit bunch and the hydrogel bunch was going to end.

## 5. Conclusions

The treatment method in this study has a certain improvement in the treatment effect of “peripheral facial paralysis” in the recovery period and has a good performance in clinical application. In this study, traditional acupuncture treatment was used as the basic treatment. By comparing the clinical efficacy of nerve repair combined with acupuncture in the treatment of “peripheral facial paralysis” during the recovery period, the results of this project can be summarized as follows: The treatment effect of “facial paralysis” during the recovery period has been improved to a certain extent, and it has a better performance in clinical application. By comparing the results of 4 evaluation indicators displayed by several groups of patients in different treatment time periods, it can be concluded that in the treatment of “peripheral facial paralysis” during the recovery period, ordinary acupuncture is used as the basic treatment, supplemented by acupuncture and moxibustion treatment. The effect is more significant. In this trial design, the treatment group used acupuncture on the basis of the control group to treat “peripheral facial paralysis” during the recovery period. The experiment showed that *t* = 2.618, *P* = 0.019 < 0.05, indicating that there was a significant difference in the HB facial nerve grading in the treatment group before and after treatment. The method is relatively novel and has a certain degree of innovation. The results show that acupuncture therapy can not only promote local qi and blood circulation in the treatment of “peripheral facial paralysis” but also solve the problem of muscle disability left by “peripheral facial paralysis” and confirm that acupuncture can treat muscle paralysis caused by motor nerve injury. This article also uses a variety of evaluation indicators to evaluate efficacy. These indicators are the main indicators for evaluating the effect of “peripheral facial paralysis” during the recovery period. The evaluation is relatively comprehensive, and the conclusions obtained are true and reliable. Because I have certain limitations in my energy, ability, time, funding, etc., this study did not conduct a large sample survey and analysis. Therefore, the accuracy, stability, avoidance of errors, and improvement of the persuasiveness of the research results are relatively lacking. The number and types of research subjects are limited to some extent. Due to limited conditions, it is impossible to carry out laboratory collection of more information (such as blood, body immune function, etc.). The inference of sexuality has not been studied with a more scientific method. I will perfect it in my work and study in the future, hoping to contribute my own strength to acupuncture and moxibustion medicine.

## Figures and Tables

**Figure 1:** Primary culture and identification of fibroblasts.

**Figure 2:** Etching of silicon with different crystal phases in KOH.

**Figure 3:** Comparison of different treatment methods for patients with facial paralysis.

**Figure 4:** Comparison of two groups after treatment efficiency.

**Figure 5:** FDIP evaluation of the two groups at the four time nodes of T1, T2, T3, and T4.

**Figure 6:** Immunofluorescence staining of Schwann cells and fibroblasts on the 14th day of nerve repair.

**Figure 7:** Electron microscope ultrastructure of the regenerated nerve tissue proximal to the catheter 3 w after operation in the TENG group.

**Figure 8:** Observation diagram of coating preparation containing artificial nerve components obtained after implantation.

**Table 1:** Two groups before treatment in patients with H—B level of facial nerve.

Group	Number of cases	Before treatment		After treatment	
		I	II	I	II
Therapy group	30	0	1	15	9
Control group	30	0	1	11	6

**Table 2:** Two groups of treatment comparisons (*n*).

Group	Number of cases	Level 1	Level 2	Level 3	Level 4
Therapy group	20	17	3	0	0
Control group	20	18	2	0	0

**Table 3:** Comparison of the latency, amplitude, and conduction velocity of nerve regeneration in each group at 8 weeks after the operation.

Group	Incubation period (ms)	Amplitude (mV)	Conduction speed (m/s)
Group A (chitosan plus PRP)	1.90 ± 0.21	3.05 ± 0.15	22.19 ± 1.19
Group B (chitosan plus saline)	2.37 ± 0.12	1.94 ± 0.06	17.85 ± 0.28
Group C (silicone tube plus saline)	2.50 ± 0.17	1.88 ± 0.03	17.45 ± 0.39
Group D (silicone tube plus PRP)	1.90 ± 0.31	2.99 ± 0.15	22.17 ± 1.22
*F* value	46.447	157.254	44.020
*P* value	0.000	0.000	0.000

**Table 4:** Comparison of Nerve Palsy Scale scores before and after treatment.

Group	Number of cases	Before treatment	After treatment
Therapy group	34	30.29 ± 13.35	87.43 ± 18.03
Control group	34	30.88 ± 13.69	76.62 ± 22.80
*Z*		−0.321	−2.172
*P*		0.748	0.030

## Data Availability

No data were used to support this study.
